RETRACTED

# Inhibition of constitutively active Jak-Stat pathway suppresses cell growth of human T-cell leukemia virus type 1-infected T-cell lines and primary adult T-cell leukemia cells

**DOI:** 10.1186/1742-4690-3-22

**Published:** 2006-04-09

**Authors:** Mariko Tomita, Hirochika Kawakami, Jun-nosuke Uchihara, Taeko Okudaira, Masato Masuda, Takehiro Matsuda, Yuetsu Tanaka, Kazuiku Ohshiro, Naoki Mori

**Affiliations:** 1 Division of Molecular Virology and Oncology, Graduate School of Medicine, University of the Ryukyus, 207 Uehara, Nishihara, Okinawa 903-0215, Japan; 2 Division of Endocrinology and Metabolism, Faculty of Medicine, University of the Ryukyus, 207 Uehara, Nishihara, Okinawa 903-0215, Japan; 3 Division of Child Health and Welfare, Faculty of Medicine, University of the Ryukyus, 207 Uehara, Nishihara, Okinawa 903-0215, Japan; 4 Division of Immunology, Faculty of Medicine, University of the Ryukyus, 207 Uehara, Nishihara, Okinawa 903-0215, Japan; 5 Department of Internal Medicine, Naha Prefectural Hospital, 1-3-1 Yogi, Naha, Okinawa 902-8531, Japan

## Abstract

**Background:**

Human T-cell leukemia virus type 1 (HTLV-1), the etiologic agent for adult T-cell leukemia (ATL), induces cytokine-independent proliferation of T-cells, associated with the acquisition of constitutive activation of Janus kinases (Jak) and signal transducers and activators of transcription (Stat) proteins. Our purposes in this study were to determine whether activation of Jak-Stat pathway is responsible for the proliferation and survival of ATL cells, and to explore mechanisms by which inhibition of Jak-Stat pathway kills ATL cells.

**Results:**

Constitutive activation of Stat3 and Stat5 was observed in HTLV-1-infected T-cell lines and primary ATL cells, but not in HTLV-1-negative T-cell lines. Using AG490, a Jak-specific inhibitor, we demonstrated that the activation of Stat3 and Stat5 was mediated by the constitutive phosphorylation of Jak proteins. AG490 inhibited the growth of HTLV-1-infected T-cell lines and primary ATL cells by inducing G_1 _cell-cycle arrest mediated by altering the expression of cyclin D2, Cdk4, p53, p21, Pim-1 and c-Myc, and by apoptosis mediated by the reduced expression of c-IAP2, XIAP, survivin and Bcl-2. Importantly, AG490 did not inhibit the growth of normal peripheral blood mononuclear cells.

**Conclusion:**

Our results indicate that activation of Jak-Stat pathway is responsible for the proliferation and survival of ATL cells. Inhibition of this pathway may provide a new approach for the treatment of ATL.

## Background

Adult T-cell leukemia (ATL) is an aggressive lymphoproliferative disorder that occurs in individuals infected with human T-cell leukemia virus type 1 (HTLV-1) [1-3]. HTLV-1 causes ATL in 3–5% of infected individuals after a long latent period of 40–60 years [4]. The prognosis of ATL patients remains poor with a median survival time of 13 months in aggressive cases [5]. The poor prognosis of ATL patients is partly due to the innate resistance of HTLV-1-infected T-cells to apoptosis and thus to conventional chemotherapy regimens. Therefore, there is a critical need for new ATL therapies with improved efficacy over current treatments.

RETRACTED

High expression of the interleukin-2 receptor α chain (IL-2Rα) is a common feature of ATL cells and HTLV-1-infected T-cell lines [6]. One of the well-documented signalling pathways mediated by IL-2R is Janus kinase (Jak)-Signal transducers and activators of transcription (Stat) [7]. Jak proteins transduce signals by phosphorylating Stat proteins, which in turn dimerize and translocate to the nucleus to activate the expression of genes necessary for cell proliferation and differentiation [8]. Abnormal activation of Stat proteins is a common characteristic found in various human tumor cell lines and human tumors including leukemia and lymphoma [9-11]. Constitutive activation of the IL-2R-Jak/Stat signalling pathway correlates with IL-2 independence of HTLV-1-transformed cell lines [12]. Constitutive Jak1, Jak3, Stat1, Stat3 and Stat5 activation was observed in HTLV-1-infected T-cell lines [13]. Similarly, an *in vitro *study with uncultured leukemic cells from HTLV-1 seropositive patients with ATL also displayed constitutive activation of Jak3, Stat1, Stat3 and Stat5 [14]. These results suggest that activation of the IL-2R signalling pathway mediated by Jak-Stat may play a key role in transformation by HTLV-1. However, a causal relationship between carcinogenesis and activation of the Jak-Stat pathway in ATL has not been established, and it is not clear whether disruption of this pathway could reverse the phenotypic condition of HTLV-1-infected T-cells.

AG490 is a recent addition to the synthetically derived tyrphostin family of tyrosine kinase inhibitors. Tyrphostins were designed on the basis of tyrosine and erbstatin and were all benzene malonitriles, many of which are substrate competitive but non-competitive inhibitors with respect to adenosine triphosphate [15]. AG490 selectively inhibits Jak family kinases but has no effect on other lymphocyte tyrosine kinases, including Lck, Lyn, Btk, Syk and Src [16,17]. Systemic administration of AG490 in SCID mice with disseminated human leukemic cells dependent on Jak2 for survival resulted in tumor cell apoptosis leading to complete tumor regression [16]. However, it has been reported that AG490 blocks the phosphorylation of Stat5 and Jak3, and DNA-binding activity of Stat5 of HTLV-1-transformed T-cell lines, but it fails to disrupt the growth of these leukemic cells [18]. In the present study, we evaluated the anti-tumor efficacy of AG490 against ATL and found that AG490 inhibited the growth of HTLV-1-infected T-cell lines and primary ATL cells, but not that of normal peripheral blood mononuclear cells (PBMCs). Furthermore, we investigated the possible mechanisms involved in such *in vitro *growth-inhibitory effect. Our findings suggested that activation of Jak-Stat signalling pathway is responsible for ATL cell proliferation and survival.

RETRACTED

## Results

### Constitutive tyrosine phosphorylation of Stat3 and Stat5 in HTLV-1-infected T-cell lines

We first examined HTLV-1-infected T-cell lines [MT-2, HUT-102 and ED-40515(-)] for the phosphorylation status of Stat3 and Stat5. All HTLV-1-infected T-cell lines displayed constitutive phosphorylation of Stat3 (Figure 1A, top panel). Constitutive phosphorylation of Stat5 was observed in MT-2 and HUT-102 (Figure 1A, third panel). In contrast, phosphorylation of Stat3 and Stat5 was not observed in HTLV-1-negative T-cell lines (Jurkat, MOLT-4 and CCRF-CEM) (Figure 1A, top and third panels), although the expression of Stat3 and Stat5 was detected in all cell lines (Figure 1A, second and forth panels). MT-2 and HUT-102 highly express HTLV-1 viral proteins, whereas ED-40515(-), a T-cell line of leukemic cell origin established from a patient with ATL, expresses little HTLV-1 viral proteins. For example, HTLV-1 transforming protein Tax was detected in MT-2 and HUT-102, but not in ED-40515(-) and all HTLV-1-negative T-cell lines (Figure 1A, second panel from the bottom). Because hypermethylation of 5' HTLV-1 long terminal repeat in ATL derived cell lines and ATL cells silenced the viral gene expression [19], ED-40515(-) cells did not express significant levels of Tax protein. These results suggested that constitutive phosphorylation of Stat3 and Stat5 seems to depend on HTLV-1 infection, but not on the expression of HTLV-1 Tax protein.

**Figure 1:** **Constitutive activation of Stat3 and Stat5 in HTLV-1-infected T-cell lines**. (A) Western blot analysis of cellular lysates prepared from three HTLV-1-negative [HTLV-1 (-)] and three HTLV-1-infected [HTLV-1 (+)] T-cell lines. The blots were probed with anti-phospho-Stat3, anti-Stat3, anti-phospho-Stat5, anti-Stat5 and anti-Tax. Amounts of actin are shown as loading controls. (B) Stat-DNA binding activities in HTLV-1-negative and HTLV-1-infected T-cell lines were detected by EMSA using SIE or β-casein probe. Arrows indicate specific protein-DNA complexes. NS indicates non-specific bands. (C) Competition assay was performed with nuclear extracts of HTLV-1-infected cell lines using 100-fold excess of unlabeled wild type (W) or mutant (M) oligonucleotide as a competitor (upper panels: SIE, lower panels: β-casein). (D and E) Involvement of Stat3 and Stat5 in the formation of SIE- (D) and β-casein- (E) binding complexes in HTLV-1-infected T-cell lines. EMSA was performed with nuclear extracts of the indicated cell lines either in the absence (-) or presence of a specific Stat antibody (αStat: anti-Stat1, Stat2, Stat3, Stat4 and Stat5 antibodies). The supershifted complexes are indicated by arrowheads.

RETRACTED

### Constitutive activation of Stat3- and Stat5-DNA binding activity in HTLV-1-infected T-cell lines

Electrophoretic mobility shift assay (EMSA) was performed to analyze Stat-DNA binding activity of HTLV-1-infected T-cell lines using two different Stat-consensus sequences from the c-*fos *gene promoter [*sis*-inducible element (SIE)] and from the β-*casein *gene promoter (β-casein) (Figure 1B). Both SIE- and β-casein-binding activities were detected in the nuclear extracts of MT-2 and HUT-102 cells. SIE- but not β-casein-binding activity was detected in extracts of ED-40515(-) cells. In contrast, no significant DNA binding activity of SIE or β-casein was detected in extracts of HTLV-1-negative T-cell lines. Competition assays showed that the observed protein-DNA complexes were specific for SIE or β-casein (Figures 1C). The SIE-binding protein complexes from MT-2, HUT-102 and ED-40515(-) cells included Stat3, since the complex was supershifted by specific antibody for Stat3 (Figure 1D). The β-casein-binding protein complexes from MT-2 and HUT-102 cells included Stat5 (Figure 1E, upper panels). Stat1, Stat2 and Stat4 specific antibodies did not influence the formation of both SIE- and β-casein-complexes in any cell lines (Figures 1D and 1E). These results indicate that constitutive phosphorylation of Stat3 and Stat5 correlates with their DNA binding activities in HTLV-1-infected T-cell lines.

### Tax is not responsible for the induction of Stat3 and Stat5 phosphorylation in T-cells

We next examined whether HTLV-1 Tax protein alters the phosphorylation status of Stat3 and Stat5. Tax-inducible T-cell line, JPX-9 expressed Tax 10 h after addition of CdCl_2 _and the expression persisted until 72 h after treatment (Figure 2, second panel from the bottom, lanes 4–7). Although Stat3 and Stat5 were consistently expressed in JPX-9 cells even after CdCl_2 _treatment, phosphorylated Stat3 and Stat5 were not detected in these cells (Figure 2, first and third panels). These results suggest that Tax is not involved in the induction of Stat3 and Stat5 phosphorylation in T-cells.

RETRACTED

**Figure 2:** **HTLV-1 Tax does not involve in phosphorylation of Stat3 and Stat5**. Cell lysates were prepared from CdCl_2_-treated JPX-9 cells at the indicated time points (lanes 1–7) and untreated MT-2 cells (lane 8: as a positive control). The expression of phospho-Stat3, Stat3, phospho-Stat5, Stat5 and Tax (arrow) was analyzed by Western blot. Actin expression served as a loading control.

### AG490 reduces constitutive activation of Stat3 and Stat5 through inhibition of Jak kinases in HTLV-1-infected T-cell lines

The regulation of phosphorylation of Stat3 and Stat5 by Jak kinases was investigated with Jak selective inhibitor, AG490. AG490 reduced constitutive phosphorylation in Stat3 [MT-2, HUT-102 and ED-40515(-)] and Stat5 (MT-2 and HUT-102) in a dose-dependent manner (Figures 3A and 3B). AG490 also suppressed constitutive phosphorylation of Stat3 and Stat5 in freshly isolated ATL cells (Figure 3C). Constitutive phosphorylation of Jak1, Jak2 and Jak3 was observed in MT-2 and HUT-102 cells, and treatment of these cells with increasing concentrations of AG490 resulted in significant inhibition of phosphorylation of Jak1, Jak2 and Jak3 (Figure 3D). Constitutive phosphorylation of Jak2 but not Jak1 and Jak3 was detected in ED-40515(-) cells and treatment with AG490 inhibited phosphorylation of Jak2 in ED-40515(-) cells (Figure 3D). AG490 did not affect on phosphorylation status of glycogen synthase kinase-3β (GSK-3β) that is not regulated by Jak-Stat pathway (Figure 3E), suggesting that effect of AG490 is specific for Jak-Stat pathway. To determine whether AG490 inhibits DNA binding activity of Stat3 and Stat5 in HTLV-1-infected T-cell lines, we treated the cells with 50 μM AG490 for 24 h and performed EMSA (Figure 3F). AG490 decreased SIE- [MT-2, HUT-102 and ED-40515(-)] and β-casein- (MT-2 and HUT-102) DNA binding activity of HTLV-1-infected T-cell lines. These results suggest that AG490 reduces the constitutive activation of Stat3 and Stat5 by inhibiting three Jak kinases in HTLV-1-infected T-cell lines.

**Figure 3:** **AG490 inhibits constitutive activation of Jak and Stat in HTLV-1-infected T-cell lines and primary ATL cells**. (A and B) HTLV-1-infected T-cell lines were treated with increasing concentrations of AG490 for 24 h. (C) Primary ATL cells were treated with (+) or without (-) 50 μM AG490 for 24 h. Phosphorylation status of Stat3 and Stat5 was assessed by Western blot analysis. (D) HTLV-1-infected T-cell lines were treated with increasing concentrations of AG490 for 24 h. Phosphorylation status of Jak1, Jak2 and Jak3 were assessed by Western blot analysis. (E) AG490 does not affect phosphorylation of other phosphor-protein that is not regulated by Jak-Stat pathway. HTLV-1-infected T-cell lines were treated with (+) or without (-) 50 μM AG490 for 24 h. Phosphorylation status of GSK-3β was assessed by Western blot analysis. (F) AG490 inhibits constitutive Stat3- and Stat5-DNA binding in HTLV-1-infected T-cell lines. Nuclear extracts were isolated from HTLV-1-infected T-cell lines treated with (+) or without (-) 50 μM AG490 for 24 h. Stat-DNA binding activity was assessed by EMSA using SIE or β-casein probe.

RETRACTED

### AG490 inhibits the cell growth of HTLV-1-infected T-cell lines and primary ATL cells

Next we examined the effect of AG490 on the growth of HTLV-1-infected T-cell lines and primary ATL cells. HTLV-1-infected T-cell lines were treated with different concentration of AG490 (0, 25 or 50 μM) and cell numbers were counted 24 and 48 h after treatment. AG490 suppressed the growth of HTLV-1-infected T-cell lines in a dose and time dependent manner (Figure 4A). The antiproliferative effects of AG490 against primary ATL cells and PBMCs from healthy donors were measured by WST-8 method (Cell Counting Kit-8; Wako Chemical, Osaka, Japan) based on the MTT assay as described previously [20]. Cell viability was determined as percentage of the control (without AG490). AG490 also inhibited the growth of PBMCs from ATL patients (ATL #1–7 in Figure 4B). In comparison, the cell growth inhibitory effect on PBMCs from healthy donors was weak (Normal #1–3 in Figure 4B). These findings indicate that AG490 inhibits the growth of cells infected with HTLV-1 but not that of uninfected PBMCs.

**Figure 4:** **AG490 reduces cell growth of HTLV-1-infected T-cell lines and primary ATL cells**. (A) HTLV-1-infected T-cell lines (5 × 10^4^/mL) were treated with 0, 25 or 50 μM AG490 for 24 or 48 h. Cell numbers were counted in triplicate by Trypan blue dye exclusion method. Data are expressed as the mean values of viable cell numbers. (B) Primary ATL cells from seven patients (ATL #1–7) and PBMCs from three healthy donors (Normal #1–3) were treated with 0, 25 or 50 μM AG490 for 48 h. Cell growth was assessed by the WST-8 method. Data are expressed as the percentages of control (untreated cells). (C) Cell-cycle analysis of HTLV-1-infected T-cell lines treated with AG490. Cells were treated in the absence (-) or presence (+) of 25 μM AG490 for 24 h. DNA content was analyzed by flow cytometry with propidium iodide staining. G_1_, S and G_2_/M indicate the stages of the cell-cycle. Data represent mean percentages of cells at each cell-cycle from three independent experiments. (D) Induction of apoptosis in HTLV-1-infected T-cell lines by AG490. Cells were treated in the absence (open bar) or presence (solid bar) of 50 μM AG490 for 48 h and stained with Annexin-V. Apoptosis was analyzed by flow cytometry. Data represent mean percentages of apoptotic cells from three independent experiments.

RETRACTED

### AG490 induces cell-cycle arrest and apoptosis of HTLV-1-infected T-cell lines

We then investigated the effect of AG490 on cell-cycle distribution in HTLV-1-infected T-cell lines (Figure 4C). Cells were treated with 25 μM AG490 for 24 h. Twenty-five μM AG490 inhibited cell-cycle progression, as demonstrated by the increased proportion of cells in G_1 _phase [MT-2: from 52% to 72%; HUT-102: from 51% to 83%; ED-40515(-): from 35% to 44%] and decreased percentage of cells in S phase [MT-2: from 36% to 18%; HUT-102: from 36% to 8%; ED-40515(-): from 51% to 43%], indicating G_1 _cell-cycle arrest. The effect of AG490 on apoptosis was examined by the Annexin-V method. Annexin-V binding reveals the phosphatidylserine molecules have been flipped out from the inner to the outer cell surface during apoptosis. Cells were treated with 50 μM AG490 for 48 h. AG490 increased the proportion of cells positive for Annexin-V in all cell lines (Figure 4D), indicating the increased apoptosis of AG490-treated cells. Thus, AG490 is both anti-proliferative and pro-apoptotic in HTLV-1-infected T-cell lines.

### Expression of cell-cycle associated genes in AG490-treated HTLV-1-infected T-cell lines and ATL cells

We next examined whether AG490 induces G_1 _cell-cycle arrest by modulating the expression of G_1 _cyclins, cyclin D1 and cyclin D2, which are associated with cell-cycle progression from G_1 _to S phase. AG490 decreased cyclin D2 expression, however, the expression of cyclin D1 was almost unchanged (Figure 5A). Cell-cycle progression from G_1 _to S phase is also regulated by G_1 _cyclin-dependent kinases; Cdk4 and Cdk6, which bind and activate the cyclin D. AG490 inhibited the expression of Cdk4 in a dose-dependent manner but not that of Cdk6 protein (Figure 5A). These results suggest that AG490 induces G_1 _arrest by reducing the expression of cyclin D2 and Cdk4, which regulate the G_1_-S transition. The p53/p21 pathway also plays a critical role in regulating the G_1_-S transition. We examined the effects of AG490 on p53 and p21 levels in HTLV-1-infected T-cell lines. Expression of p53 protein was increased in AG490 treated MT-2 and HUT-102 cells. In contrast, p53 protein was almost undetectable in ED-40515(-) cells and remained unchanged in AG490-treated cells. p21 was induced in MT-2 and HUT-102 cells and remained undetectable in ED-40515(-) cells. These results indicate that p21 activation can also contribute to AG490-induced G_1 _arrest in p53-competent cells. AG490-treated ED-40515(-) cells did not induce G_1 _arrest as much as MT-2 and HUT-102 cells (Figure 4D). This might be due to absence of p53 and p21 proteins in AG490-treated ED-40515(-) cells. Cell-cycle progression from G_1 _to S phase is also regulated by Serin/Threonin kinase Pim-1 and c-Myc through Cdc25A activation [21,22]. *pim-1 *and c*-myc *genes are both direct targets of Stat [23,24]. AG490 decreased the expression of these proteins in all HTLV-1-infected T-cell lines (Figure 5A). AG490 also reduced the expression of cyclin D2 and increased the expression of p53 in freshly isolated ATL cells (Figure 5B). However, other proteins that were altered by AG490 in HTLV-1-infected T-cell lines were undetectable and AG490 did not change the expression of these genes in primary ATL cells (data not shown).

RETRACTED

**Figure 5:** **Effects of AG490 on the expression of cell-cycle associated proteins**. HTLV-1-infected T-cell lines were treated with increasing concentrations of AG490 for 24 h. Amounts of cyclin D1, cyclin D2, Cdk4, Cdk6, p53, p21, Pim-1 and c-Myc were determined by Western blot analysis. (B) Primary ATL cells were treated with (+) or without (-) 50 μM AG490 for 24 h. The expression of cyclin D2 and p53 was assessed by Western blot analysis. The amount of actin is shown as a loading control.

### Expression of anti-apoptotic genes in AG490-treated HTLV-1-infected T-cell lines and ATL cells

We also examined the effects of AG490 on the expression of IAP and Bcl-2 family members, which determine the response to apoptotic stimuli. AG490 significantly altered the expression of XIAP and survivin, which are Stat-regulated genes [25,26], but not that of Bcl-x_L _protein in all tested cell lines (Figure 6A). Downregulation of Bcl-2 expression by AG490 was only noted in HUT-102 cells. The expression of c-IAP2 was downregulated in HUT-102 and ED-40515(-), but not in MT-2 cells. These results indicated that AG490-induced apoptosis of HTLV-1-infected T-cells is mediated by downregulation of c-IAP2, XIAP, survivin and Bcl-2 expression. AG490 reduced the expression of all these genes in freshly isolated ATL cells (Figure 6B). Bcl-2 protein was undetectable in primary ATL cells (data not shown). Cyclin D2 [27,28], Cdk4 [29], XIAP [30] and survivin [31] are Tax-responsive genes, therefore, we also examined the level of Tax expression in these cells. AG490 did not alter Tax protein levels in MT-2 and HUT-102 cells (Figure 6A). Tax protein remained at undetectable levels in ED-40515(-) and primary ATL cells after AG490 treatment (Figures 6A and 6B). Therefore, the altered expression of cyclin D2, Cdk4, XIAP and survivin was not attributable to Tax downregulation. We also examined whether AG490 could change the expression levels of other viral proteins. The expression levels of HTLV-1 envelope 46 kDa glycoprotein (gp46) and 19 kDa core protein (p19) were not changed by AG490 treatment in HUT-102 cells (Figure 6C), suggesting that the AG490 does not drop the virus levels in these cells and the effects of AG490 on these cells are not due to downregulation of viral proteins.

RETRACTED

**Figure 6:** **Effects of AG490 on the expression of anti-apoptotic proteins**. (A) HTLV-1-infected T-cell lines were treated with increasing concentrations of AG490 for 24 h. Amounts of c-IAP-2, XIAP, survivin, Bcl-2, Bcl-x_L _and Tax were determined by Western blot analysis. (B) Primary ATL cells were treated with (+) or without (-) 50 μM AG490 for 24 h. The expression of c-IAP2, XIAP, survivin and Tax was assessed by Western blot analysis. (C) HUT-102 cells were treated with (+) or without (-) 50 μM AG490 for 24 h. The expression of HTLV-1 viral proteins, envelope glycoprotein gp46 and p19 core protein was assessed by Western blot analysis. The amount of actin is shown as a loading control.

## Discussion

In this study, we demonstrated that Stat3 and Stat5 are constitutively activated in HTLV-1-infected T-cell lines and primary ATL cells, but not in HTLV-1-negative T-cell lines. Using AG490, a Jak-specific inhibitor, we showed that the activation of Stat3 and Stat5 is mediated by the constitutive phosphorylation of Jak proteins. Furthermore, we showed that AG490 inhibits the growth of HTLV-1-infected T-cell lines and primary ATL cells by inducing G_1 _cell-cycle arrest and apoptosis, but not that of normal PBMCs. Our results indicate that constitutive activation of Jak-Stat is responsible for the proliferation and survival of ATL cells.

The mechanism for the constitutive activation of Jak-Stat after HTLV-1 infection is still unclear. HTLV-1 transforming protein Tax is considered to play a critical role in leukemogenesis and development of ATL. However, our data showed no correlation between Stat activation and Tax protein expression in HTLV-1-infected T-cell lines. Previous reports are consistent with our data in their lack of support for the involvement of Tax or the autocrine production of IL-2 or IL-15 in Stat-activation of HTLV-1-infected T-cell lines and primary ATL cells [12,14]. Expression of Stat5 mRNA is induced by HTLV-1 Tax using JPX-9 cells [32]. Using this cell line, we showed that Tax induced neither the expression nor the phosphorylation of Stat3 and Stat5 proteins. A T-cell line denoted Tax, in which a herpes samiri-based vector drives *Tax *gene expression, does not exhibit constitutive Stat binding activity [12]. We also showed that ATL-derived T-cell line, ED-40515(-) and primary ATL cells which did not express Tax protein at detectable level, expressed Stat proteins in the phosphorylated form. It should be noted that the leukemic cells *in vivo *generally do not express Tax by several mechanisms [33]. Thus, it is unlikely that Tax is involved in the induction or activation of Stat proteins or represents a target of anti-ATL drugs. Previously, Nicot and colleagues [34] reported that the p12^I ^protein, encoded by the pX open reading frame I of HTLV-1, binds to the IL-2R β chain, resulting in activation of Stat5 through Jak1 and Jak3 activation. However, the mechanisms for the Jak2 activation in HTLV-1-infected T-cells are not elucidated.

RETRACTED

Our data demonstrating that inhibition of Stat activity led to apoptosis in HTLV-1-infected T-cell lines and primary ATL cells are in line with a previous study reporting induction of apoptosis by ectopic expression of a dominant-negative form of Stat5 in MT-2 cells [25]. Our data of a weaker effect of AG490 on the growth of normal PBMCs than that of ATL cells were consistent with a previous report showing that AG490 has no significant effect on the growth of normal B and T cells *in vitro *[16]. In contrast to our data, Kirken and colleagues [18] reported that although AG490 blocks the phosphorylation of Stat5 and Jak3, and DNA-binding activity of Stat5 of HTLV-1-transformed T-cell lines, MT-2 and HUT-102, it fails to disrupt the growth of these leukemic cells. Although we used lower concentration of AG490 (50 μM Max.) than this group (100 μM Max.), we observed a dose-dependent inhibition of cell growth in these cells by AG490. The precise reason for these differences is not clear, however, we cannot exclude the possibility that these differences could be attributable to variations in experimental conditions such as serum concentration (1% vs. 10%) in tissue culture medium. Perhaps for AG490 mediated growth inhibitory effect in HTLV-1-infected T-cell lines and ATL cells, active protein synthesis is required.

Previous study suggested that AG490 is a Jak2-specific inhibitor and blocks leukemic cell growth of acute lymphoblastic leukemia [16]. Our data showed that AG490 also inhibited phosphorylation of Jak1 and Jak3 of MT-2 and HUT-102. Thus, three constitutively phosphorylated Jak proteins in HTLV-1-infected T-cell lines were inhibited by AG490. These results are consistent with recent studies reporting that AG490 inhibits Jak1 activated by IL-6 in myeloma cells or IL-2-induced Jak3 activity in an IL-2-dependent T-cell line [17,35], suggesting that the aforementioned three Jak proteins share AG490 sensitivity. Interestingly, AG490 does not affect other lymphocyte tyrosine kinases [16]. This may also account for the fact that AG490 is well-tolerated in mice [16,36].

RETRACTED

## Conclusion

We have demonstrated that constitutive activation of Jak-Stat is responsible for the proliferation and survival of ATL cells. Previously we showed that NF-κB pathway is constitutively activated in HTLV-1-infected T-cell lines and primary ATL cells [37] and inhibition of this pathway suppresses the growth of these cells [38,39]. In addition to NF-κB pathway, our findings in this study indicate that inhibition of the Jak-Stat pathway offers a new approach for ATL treatment. Furthermore, AG490 kinase inhibitor is well tolerated *in vivo*, and thus presents a useful agent for this novel anti-ATL therapeutic approach.

## Methods

### Cell lines

The HTLV-1-uninfected T-cell leukemia cell lines; Jurkat, MOLT-4, CCRF-CEM and HTLV-1-infected T-cell lines; MT-2 [40], HUT-102 [1] and ED-40515(-) [41] [HUT-102 was a generous gift from the Fujisaki Cell Center, Hayashibara Biomedical Laboratories, Okayama, Japan, ED-40515(-) was from Dr. M. Maeda, Kyoto University, Kyoto, Japan] were maintained in RPMI 1640 medium supplemented with 10% heat-inactivated fetal bovine serum, 50 U/ml penicillin and 50 μg/ml streptomycin (Sigma-Aldrich, St. Louis, MO) at 37°C in 5% CO_2_. MT-2 is an HTLV-1-transformed T-cell line, established by an *in vitro *coculture protocol. The clonal origin of HUT-102 was not determined. ED-40515(-) is a leukemia T-cell line derived from a patient with ATL. JPX-9 (kindly provided by Dr. M. Nakamura, Tokyo Medical and Dental University, Tokyo, Japan) is a subclone of Jurkat cells expressing Tax under the control of the metallothionein promoter [42]. Expression of Tax was induced by addition of CdCl_2 _to a final concentration of 20 μM.

### Reagents

AG490 was purchased from Calbiochem (La Jolla, CA). The anti-Tax (Lt-4), anti-gp46 (REY-7) and anti-p19 (GIN-7) antibodies were described previously [43-45]. The anti-Stat3, anti-phospho-Stat3 (Tyr705), anti-phospho-Stat5 (Tyr694) and anti-phospho-GSK-3β (Ser9) antibodies were purchased from Cell Signaling Technology (Beverly, MA). The anti-phospho-Jak1 (Tyr 1022/Tyr 1023), anti-phospho-Jak2 (Tyr 1007/Tyr 1008), anti-phospho-Jak3 (Try980), anti-cyclin D2, anti-Pim-1, anti-survivin and anti-c-IAP2 antibodies were purchased from Santa Cruz Biotechnology (Santa Cruz, CA). The anti-cyclin D1 and anti-XIAP antibodies were purchased from Medical & Biological Laboratories (Nagoya, Japan). The anti-Cdk4, anti-Cdk6, anti-p53, anti-p21, anti-c-Myc, anti-Bcl-2 and anti-actin antibodies were from NeoMarkers (Fremont, CA). The anti-Stat5 and anti-Bcl-x_L _antibodies were from BD transduction Laboratories (San Jose, CA). Horseradish-peroxidase-conjugated secondary antibodies were purchased from Amersham Biosciences (Piscataway, NJ).

RETRACTED

### Western blot analysis

Western blot analysis was performed as described previously [46]. In brief, whole cell lysates were subjected to SDS-PAGE and electroblotted onto polyvinylidene difluoride membranes (Millipore, Billerica, MA), and then analyzed for immunoreactivity with the appropriate primary and secondary antibodies as indicated in the figures. Reaction products were visualized using Enhanced Chemiluminescence reagent, according to the instructions provided by the manufacturer (Amersham Pharmacia, Uppsala, Sweden).

### EMSA

Nuclear extracts were prepared from AG490-treated and untreated cells and Stat3- or Stat5-DNA binding activity was analyzed by EMSA as described previously [47,48]. The probes or competitors used were prepared by annealing the following sense and antisense synthetic oligonucleotides: Stat3 consensus binding motif (SIE) derived from c-*fos *promoter 5'-gatcGACATTTCCCGTAAATCG-3', SIE mutant 5'-gatcGACATTTCCCGTCCCGCG-3', Stat5 consensus binding motif (β-casein) derived from β-*casein *promoter 5'-gatcAGATTTCTAGGAATTCAAATC-3' and β-casein mutant 5'-gatcAGATTTAGTTTAATTCAAATC-3'. To identify Stat proteins in the DNA-protein complex revealed by EMSA, we used specific antibodies for various Stat family proteins including Stat1, Stat2, Stat3, Stat4 and Stat5 (Santa Cruz Biotechnology), to elicit a supershift DNA-protein complex formation.

### Patient samples

PBMCs from three healthy volunteers (Normal #1–3) or patients with the acute (ATL #1–4, 6 and 7) or chronic (ATL #5) type of ATL were analyzed. The diagnosis of ATL was based on clinical features, hematological characteristics, presence of serum antibodies to ATL-associated antigens and presence of HTLV-1 proviral genome in DNA from leukemic cells. PBMCs were isolated by Ficoll/Hypaque (Pharmacia LKB, Piscataway, NJ) using density gradient centrifugation. Each patient had more than 90% leukemic cells in the blood at the time of analysis. The study protocol was approved by the Human Ethics Review Committee of University of the Ryukyus, and a signed consent form was obtained from each subject.

### Assays for cellular proliferation

The antiproliferative effects of AG490 against HTLV-1-infected T-cell lines were measured by the Trypan blue dye exclusion method. The 5 × 10^4 ^cells were incubated in the presence of 0, 25 or 50 μM AG490 in a final volume of 1 mL at 37°C. The cell numbers were counted by the Trypan blue dye exclusion method after 24 and 48 h treatment. The antiproliferative effects of AG490 against primary ATL cells and PBMCs from healthy donors were measured by WST-8 method (Cell Counting Kit-8; Wako Chemical, Osaka, Japan) based on the MTT assay as described previously [20]. Briefly, the 1 × 10^5 ^cells were incubated in triplicate in 96-well microculture plates in the presence of 0, 25 or 50 μM AG490 in a final volume of 0.1 ml for 48 h at 37°C. Thereafter, 5 μl Cell Counting Kit-8 solution [5 mM WST-8, 0.2 mM 1-Methoxy PMS (5-methylphenazinium methylsulfate) and 150 mM NaCl] was added, and the cells were further incubated for another 4 h. The number of surviving cells was measured by a 96-well multiscanner autoreader at optical density of 450 nm. Cell viability was determined as percentage of the control (without AG490).

RETRACTED

### Cell-cycle analysis

Cells were plated at a density of 1 × 10^5^/ml in 60-mm tissue culture dish. Twelve hours after plating, cells were exposed to 25 μM AG490 for 24 h. Cell-cycle analysis was performed with the CycleTEST PLUS DNA reagent kit (Becton Dickinson, San Jose, CA). Briefly, cells were washed with a buffer solution containing sodium citrate, sucrose and dimethyl sulfoxide, suspended in a solution containing RNase A, and stained with 125 μg/ml propidium iodide for 10 min. Cell suspensions were analyzed on a FACS Calibur (Becton Dickinson) using CellQuest. The cell population at each cell-cycle phase was determined with ModiFit software.

### Assays for apoptosis

Cells were plated at a density of 1 × 10^5^/ml in 60-mm tissue culture dish. Twelve hours after plating, cells were exposed to 50 μM AG490 for 48 h. Apoptosis was quantified by staining with Annexin-V-Fluos (Roche Diagnostics, Mannheim, Germany) according to the instructions supplied by the manufacturer. Cells were analyzed on a FACS Calibur using CellQuest.

## Competing interests

The author(s) declare that they have no competing interests.

## Authors' contributions

MT contributed to the concept and design, interpreted and analyzed the data, provided drafting of the article, provided critical revisions and important intellectual content, collected and assembled the data. HK, JU, TO and TM collected and assembled the data. MM, YT and KO provided study materials and critical revisions and important intellectual content. NM contributed to the concept and design, provided critical revisions and important intellectual content, obtained a funding source, provided administrative support. All authors read and approved the final manuscript.

## References

[B1] Poiesz BJ, Ruscetti FW, Gazdar AF, Bunn PA, Minna JD, Gallo RC (1980). Detection and isolation of type C retrovirus particles from fresh and cultured lymphocytes of a patient with cutaneous T-cell lymphoma. Proc Natl Acad Sci U S A.

RETRACTED

[B2] Hinuma Y, Nagata K, Hanaoka M, Nakai M, Matsumoto T, Kinoshita KI, Shirakawa S, Miyoshi I (1981). Adult T-cell leukemia: antigen in an ATL cell line and detection of antibodies to the antigen in human sera. Proc Natl Acad Sci U S A.

[B3] Yoshida M, Miyoshi I, Hinuma Y (1982). Isolation and characterization of retrovirus from cell lines of human adult T-cell leukemia and its implication in the disease. Proc Natl Acad Sci U S A.

[B4] Tajima K (1990). The 4th nation-wide study of adult T-cell leukemia/lymphoma (ATL) in Japan: estimates of risk of ATL and its geographical and clinical features. The T- and B-cell Malignancy Study Group. Int J Cancer.

[B5] Yamada Y, Tomonaga M, Fukuda H, Hanada S, Utsunomiya A, Tara M, Sano M, Ikeda S, Takatsuki K, Kozuru M, Araki K, Kawano F, Niimi M, Tobinai K, Hotta T, Shimoyama M (2001). A new G-CSF-supported combination chemotherapy, LSG15, for adult T-cell leukaemia-lymphoma: Japan Clinical Oncology Group Study 9303. Br J Haematol.

[B6] Franchini G (1995). Molecular mechanisms of human T-cell leukemia/lymphotropic virus type I infection. Blood.

[B7] Schindler C, Darnell JEJ (1995). Transcriptional responses to polypeptide ligands: the JAK-STAT pathway. Annu Rev Biochem.

[B8] Darnell JEJ (1997). STATs and gene regulation. Science.

[B9] Bowman T, Garcia R, Turkson J, Jove R (2000). STATs in oncogenesis. Oncogene.

[B10] Coffer PJ, Koenderman L, de Groot RP (2000). The role of STATs in myeloid differentiation and leukemia. Oncogene.

[B11] Lin TS, Mahajan S, Frank DA (2000). STAT signaling in the pathogenesis and treatment of leukemias. Oncogene.

[B12] Migone TS, Lin JX, Cereseto A, Mulloy JC, O'Shea JJ, Franchini G, Leonard WJ (1995). Constitutively activated Jak-STAT pathway in T cells transformed with HTLV-I. Science.

[B13] Mulloy JC, Migone TS, Ross TM, Ton N, Green PL, Leonard WJ, Franchini G (1998). Human and simian T-cell leukemia viruses type 2 (HTLV-2 and STLV-2pan-p) transform T cells independently of Jak/STAT activation. J Virol.

[B14] Takemoto S, Mulloy JC, Cereseto A, Migone TS, Patel BK, Matsuoka M, Yamaguchi K, Takatsuki K, Kamihira S, White JD, Leonard WJ, Waldmann T, Franchini G (1997). Proliferation of adult T cell leukemia/lymphoma cells is associated with the constitutive activation of JAK/STAT proteins. Proc Natl Acad Sci U S A.

[B15] Levitzki A (2002). Tyrosine kinases as targets for cancer therapy. Eur J Cancer.

[B16] Meydan N, Grunberger T, Dadi H, Shahar M, Arpaia E, Lapidot Z, Leeder JS, Freedman M, Cohen A, Gazit A, Levitzki A, Roifman CM (1996). Inhibition of acute lymphoblastic leukaemia by a Jak-2 inhibitor. Nature.

RETRACTED

[B17] Wang LH, Kirken RA, Erwin RA, Yu CR, Farrar WL (1999). JAK3, STAT, and MAPK signaling pathways as novel molecular targets for the tyrphostin AG-490 regulation of IL-2-mediated T cell response. J Immunol.

[B18] Kirken RA, Erwin RA, Wang L, Wang Y, Rui H, Farrar WL (2000). Functional uncoupling of the Janus kinase 3-Stat5 pathway in malignant growth of human T cell leukemia virus type 1-transformed human T cells. J Immunol.

[B19] Koiwa T, Hamano-Usami A, Ishida T, Okayama A, Yamaguchi K, Kamihira S, Watanabe T (2002). 5'-long terminal repeat-selective CpG methylation of latent human T-cell leukemia virus type 1 provirus in vitro and in vivo. J Virol.

[B20] Ishiyama M, Tominaga H, Shiga M, Sasamoto K, Ohkura Y, Ueno K (1996). A combined assay of cell viability and in vitro cytotoxicity with a highly water-soluble tetrazolium salt, neutral red and crystal violet. Biol Pharm Bull.

[B21] Rainio EM, Sandholm J, Koskinen PJ (2002). Cutting edge: Transcriptional activity of NFATc1 is enhanced by the Pim-1 kinase. J Immunol.

[B22] Galaktionov K, Chen X, Beach D (1996). Cdc25 cell-cycle phosphatase as a target of c-myc. Nature.

[B23] Borg KE, Zhang M, Hegge D, Stephen RL, Buckley DJ, Magnuson NS, Buckley AR (1999). Prolactin regulation of pim-1 expression: positive and negative promoter elements. Endocrinology.

[B24] Kiuchi N, Nakajima K, Ichiba M, Fukada T, Narimatsu M, Mizuno K, Hibi M, Hirano T (1999). STAT3 is required for the gp130-mediated full activation of the c-myc gene. J Exp Med.

[B25] Mohapatra S, Chu B, Wei S, Djeu J, Epling-Burnette PK, Loughran T, Jove R, Pledger WJ (2003). Roscovitine inhibits STAT5 activity and induces apoptosis in the human leukemia virus type 1-transformed cell line MT-2. Cancer Res.

[B26] Aoki Y, Feldman GM, Tosato G (2003). Inhibition of STAT3 signaling induces apoptosis and decreases survivin expression in primary effusion lymphoma. Blood.

[B27] Huang Y, Ohtani K, Iwanaga R, Matsumura Y, Nakamura M (2001). Direct trans-activation of the human cyclin D2 gene by the oncogene product Tax of human T-cell leukemia virus type I. Oncogene.

[B28] Mori N, Fujii M, Hinz M, Nakayama K, Yamada Y, Ikeda S, Yamasaki Y, Kashanchi F, Tanaka Y, Tomonaga M, Yamamoto N (2002). Activation of cyclin D1 and D2 promoters by human T-cell leukemia virus type I tax protein is associated with IL-2-independent growth of T cells. Int J Cancer.

[B29] Iwanaga R, Ohtani K, Hayashi T, Nakamura M (2001). Molecular mechanism of cell cycle progression induced by the oncogene product Tax of human T-cell leukemia virus type I. Oncogene.

[B30] Kawakami A, Nakashima T, Sakai H, Urayama S, Yamasaki S, Hida A, Tsuboi M, Nakamura H, Ida H, Migita K, Kawabe Y, Eguchi K (1999). Inhibition of caspase cascade by HTLV-I tax through induction of NF-κB nuclear translocation. Blood.

RETRACTED

[B31] Kawakami H, Tomita M, Matsuda T, Ohta T, Tanaka Y, Fujii M, Hatano M, Tokuhisa T, Mori N (2005). Transcriptional activation of survivin through the NF-κB pathway by human T-cell leukemia virus type I tax. Int J Cancer.

[B32] Nakamura N, Fujii M, Tsukahara T, Arai M, Ohashi T, Wakao H, Kannagi M, Yamamoto N (1999). Human T-cell leukemia virus type 1 Tax protein induces the expression of STAT1 and STAT5 genes in T-cells. Oncogene.

[B33] Matsuoka M (2005). Human T-cell leukemia virus type I (HTLV-I) infection and the onset of adult T-cell leukemia (ATL). Retrovirology.

[B34] Nicot C, Mulloy JC, Ferrari MG, Johnson JM, Fu K, Fukumoto R, Trovato R, Fullen J, Leonard WJ, Franchini G (2001). HTLV-1 p12I protein enhances STAT5 activation and decreases the interleukin-2 requirement for proliferation of primary human peripheral blood mononuclear cells. Blood.

[B35] De Vos J, Jourdan M, Tarte K, Jasmin C, Klein B (2000). JAK2 tyrosine kinase inhibitor tyrphostin AG490 downregulates the mitogen-activated protein kinase (MAPK) and signal transducer and activator of transcription (STAT) pathways and induces apoptosis in myeloma cells. Br J Haematol.

[B36] Constantin G, Laudanna C, Brocke S, Butcher EC (1999). Inhibition of experimental autoimmune encephalomyelitis by a tyrosine kinase inhibitor. J Immunol.

[B37] Mori N, Fujii M, Ikeda S, Yamada Y, Tomonaga M, Ballard DW, Yamamoto N (1999). Constitutive activation of NF-kB in primary adult T-cell leukemia cells. Blood.

[B38] Mori N, Yamada Y, Ikeda S, Yamasaki Y, Tsukasaki K, Tanaka Y, Tomonaga M, Yamamoto N, Fujii M (2002). Bay 11-7082 inhibits transcription factor NF-kB and induces apoptosis of HTLV-I-infected T-cell lines and primary adult T-cell leukemia cells. Blood.

[B39] Tomita M, Kawakami H, Uchihara JN, Okudaira T, Masuda M, Takasu N, Matsuda T, Ohta T, Tanaka Y, Ohshiro K, Mori N (2006). Curcumin (diferuloylmethane) inhibits constitutive active NF-kB, leading to suppression of cell growth of human T-cell leukemia virus type I-infected T-cell lines and primary adult T-cell leukemia cells. Int J Cancer.

[B40] Miyoshi I, Kubonishi I, Yoshimoto S, Akagi T, Ohtsuki Y, Shiraishi Y, Nagata K, Hinuma Y (1981). Type C virus particles in a cord T-cell line derived by co-cultivating normal human cord leukocytes and human leukaemic T cells. Nature.

[B41] Maeda M, Shimizu A, Ikuta K, Okamoto H, Kashihara M, Uchiyama T, Honjo T, Yodoi J (1985). Origin of human T-lymphotrophic virus I-positive T cell lines in adult T cell leukemia. Analysis of T cell receptor gene rearrangement. J Exp Med.

RETRACTED

[B42] Nagata K, Ohtani K, Nakamura M, Sugamura K (1989). Activation of endogenous c-fos proto-oncogene expression by human T- cell leukemia virus type I-encoded p40tax protein in the human T-cell line, Jurkat. J Virol.

[B43] Tanaka Y, Yoshida A, Takayama Y, Tsujimoto H, Tsujimoto A, Hayami M, Tozawa H (1990). Heterogeneity of antigen molecules recognized by anti-tax1 monoclonal antibody Lt-4 in cell lines bearing human T cell leukemia virus type I and related retroviruses. Jpn J Cancer Res.

[B44] Tanaka Y, Yasumoto M, Nyunoya H, Ogura T, Kikuchi M, Shimotohno K, Shiraki H, Kuroda N, Shida H, Tozawa H (1990). Generation and characterization of monoclonal antibodies against multiple epitopes on the C-terminal half of envelope gp46 of human T-cell leukemia virus type-I (HTLV-I). Int J Cancer.

[B45] Tanaka Y, Lee B, Inoi T, Tozawa H, Yamamoto N, Hinuma Y (1986). Antigens related to three core proteins of HTLV-I (p24, p19 and p15) and their intracellular localizations, as defined by monoclonal antibodies. Int J Cancer.

[B46] Tomita M, Choe J, Tsukazaki T, Mori N (2004). The Kaposi's sarcoma-associated herpesvirus K-bZIP protein represses transforming growth factor b signaling through interaction with CREB-binding protein. Oncogene.

[B47] Mori N, Fujii M, Iwai K, Ikeda S, Yamasaki Y, Hata T, Yamada Y, Tanaka Y, Tomonaga M, Yamamoto N (2000). Constitutive activation of transcription factor AP-1 in primary adult T-cell leukemia cells. Blood.

[B48] Mori N, Prager D (1996). Transactivation of the interleukin-1α promoter by human T-cell leukemia virus type I and type II Tax proteins. Blood.

